The article "Experimental Study on the Effect of Speed Strength Training on the Special Strikes of Chinese Female Boxers" was published in 2022. Journal: J Environ Public Health.

# Experimental Study on the Effect of Speed Strength Training on the Special Strikes of Chinese Female Boxers

**DOI:** 10.1155/2022/5912231

**Published:** 2022-07-05

**Authors:** Xiangui Bu

**Affiliations:** School of Competitive Sports, Shandong Sport University, Rizhao 276800, China

## Abstract

The aim of this study was to design a 12-week intervention experiment with a speed strength training program and conventional training to test and analyze the effects of speed strength training on punching speed, punching power, and punching effectiveness of female boxers and to provide empirical support for the targeted improvement of special striking effectiveness of female boxers. By using the experimental method, a controlled experiment was conducted with 20 athletes from the Chinese women's boxing team as the study subjects, and the targeted experimental intervention was conducted. Through experiment, speed power training had no significant effect on the improvement of basic movement ability of female boxers. In addition, speed power training could effectively improve the speed power level of athletes in the experimental group, and the speed power level of the control group was not significantly improved. Lastly, speed power training improved the punching effect of the experimental group, and the effect of the control group was not significant. Conclusion of this study includes the following: (1) speed strength training improved the speed strength level of the athletes, but it did not have a significant effect on improving basic movement ability. (2) The improvement of speed strength could improve the striking speed of female boxers, and the speed strength training also achieved good results. (3) The improvement of speed strength had a positive effect on the special striking power of female boxers. (4) Speed strength training improved the special striking effect of female boxers athletes' special hitting effect.

## 1. Introduction

With the continuous development of women's boxing techniques and tactics, women's boxing matches are becoming more and more intense, direct physical confrontation is enhanced, and the role of speed and power of special striking is becoming more and more prominent, so it is of great theoretical and practical significance to explore training methods to improve the effect of special striking of women boxers. Boxing, as a sport characterized by intense physical confrontation, has high requirements for the strength and speed qualities of athletes, and in order to be able to improve their game performance, athletes also make speed and strength a key aspect of improvement, and synchronize explosive power and reaction ability training, which can significantly improve their performance on the playing field through the effective use of technical movements. Usually, we classify boxers' strength training according to strength endurance training, maximum strength training, and speed strength training, and with the development of techniques and tactics, the impact of athletes' speed strength on the outcome of the game is becoming more and more obvious [1]. However, in the current training development process, the practice of skills still occupies the main position, and quality training has been used as an aid to skills training [2, 3]. Therefore, this article explores the importance of speed power through the study of speed power on the effect of female boxers' punching, provides theoretical support and practical proof for the research of speed power training, improves the importance of speed power for female boxers, adopts targeted training to improve speed power level, promotes the overall development of female athletes, and improves the competitive level and competition performance.

## 2. Research Objects and Methods

### 2.1. Research Subjects

In this article, 20 athletes of Chinese women's national boxing team were used as the research subjects. Among them, 8 athletes were 21 years old, 7 athletes were 22 years old, and 5 athletes were 23 years old; 5 athletes were international fitness level athletes, 9 were national fitness level athletes, and 6 were national level athletes; 7 athletes had 5–6 years of training, 9 athletes had 7–8 years of training, and 4 athletes had more than 8 years of training.

### 2.2. Research Methods

#### 2.2.1. Experimental Method

Twenty boxers from the Chinese women's boxing team were selected and divided into an experimental group with similar overall characteristics and a control group for experimental comparison study according to their age and training years. The control group used conventional training methods, while the experimental group strengthened speed strength training in their training. The experimental site was in the Training Bureau of the General Administration of Sports in Beijing. The experimental period was from September 2021 to December 2021. Through the comparative analysis of the test indexes related to the punching effect before and after the experiment, the effect of speed strength on the effect of special striking was summarized.

*(1) Experimental Principle*. In order to clarify the effect of speed strength training on the special striking effect of women's boxing, this article conducted a study using a controlled experiment with controlled variables. The 20 athletes who participated in the experiment were divided into two groups with close overall level according to the characteristics of age, sports level, and training years, which were the experimental group and the control group. In the following training, the experimental group was arranged according to the traditional training method with the addition of speed strength training, while the control group was only trained in the traditional training method, which ensured that the overall training intensity and training time were the same and ensured that the experimental variable of whether to conduct speed strength strengthening training was one, and through the comparative analysis of the test of the special hitting effect of the two groups of athletes before and after training, it was possible to draw the required conclusions [4].

*(2) Training Program*. As shown in Table 1, the athletes in the experimental group participated in training 3 times a week, including traditional strength training and speed strength strengthening training, which were the same as those in the control group. The traditional strength training was conducted using barbell, dumbbell, and other equipment, with 8–12 times per group and 1-min rest between groups, while the speed strength strengthening training included explosive training such as narrow jumping pushups, with 12–15 times per group and one-minute rest between groups. Perform preparatory activities before training and stretching exercises at the end of training to ensure full recovery of the athlete's body.

As can be seen from Table 2, the control group athletes participated in training three times a week, consistent with the experimental group athletes. In the training program of the control group, only traditional strength training was arranged without speed strength strengthening training to control the experimental variables. To ensure consistent overall training intensity, the control group athletes increased the number of sets of traditional strength training to 6 sets. Warm-up was performed before training and stretching was performed at the end of training to ensure adequate recovery of the athletes.

*(3) Test Means*. In order to clarify the athletes' basic movement ability level, the athletes' performance in deep squat, front and back split-leg squat, straight knee leg raise, shoulder joint flexibility, pushup, and rotation stability were scored [5].

In order to clarify the athletes' speed strength level, seated flat pushing solid ball and 15-s fast pushup were used as test items to record the athletes' scores in both tests [6]. In the sitting flat pushing solid ball project, the faster the athletes' palms move forward, the faster the solid ball leaves the hand, and under the condition of gravity and air resistance, the performance of the flat pushing solid ball is proportional to the speed of the athletes' palms pushing out, so the performance of this project is used as the basis for testing the athletes' speed and strength level. And in the pushup, the faster the speed strength of the athlete, the shorter the time to complete a single pushup and then be able to complete more pushups in a fixed period of time, so also the performance of the 15-s fast pushup as the basis for the evaluation of the athlete's strength level.

To clarify the level of athlete's punching speed, the Sony HDR-CX630E 4K digital camera was used to photograph the athlete's punching action and calculate the speed of punching based on the image [7]. In order to clarify the level of punching power of the athlete, a comb-shaped short-tailed 18-mm resistive pressure-sensitive sensor was used and the sensor was fixed to the boxing glove, which in turn enabled the measurement of punching power [8].

## 3. Research Results and Analysis

### 3.1. Comparison Analysis of Athletes' Basic Movement Ability before and after the Experiment

Basic movements are the basis for athletes to perform physical training and special movement skills, and in the modern training theory, insufficient basic movement ability will lead athletes to compensate for training movements through muscles and joints other than the target part of the training when performing training movements, which will lead to the long-term adverse effects of nonstandard training movements on athletes' training effects and may cause sports injuries [9, 10]. In this test, deep squats, front and back split-leg squats, straight knee leg lifts, shoulder flexibility, pushups, and rotation stability were used as the items tested, and in the test results, 3 points were recorded for being able to complete the movement according to the standard, 2 points for completing the movement under compensation, 1 point for not being able to complete the movement, and 0 points for feeling pain during the completion of the movement. No warm-up exercises were performed before the test, and three consecutive tests were conducted. If 3 points were obtained in one of the tests, the final score was 3. If none of the tests reached 3 points, the lowest score was taken. To ensure the accuracy of the test results, proper warm-up is performed before the athlete performs the test.

As shown in Table 3, it can be seen that the experimental process can slightly improve the basic movement ability of some athletes, but there is no significant difference between the experimental group and the control group, which indicates that the training of speed strength has no significant effect on the improvement of basic movement ability.

### 3.2. Comparison Analysis of Athletes' Basic Speed and Strength Indexes before and after the Experiment

In order to determine the level of athletes' basic speed strength, the athletes' speed strength level was tested before and after the experiment by using the sitting flat pushing solid ball and 15-s fast pushup items, and the changes in the athletes' speed strength-related indexes were compared before and after the experiment. The test results are shown in Table 4.

As can be seen from Table 5, in order to ensure the reasonableness of the grouping and to meet the basic requirements of the controlled experiment, the speed strength level of the athletes was tested before the experiment. The results achieved by the athletes of the experimental and control groups in the two test items of sitting flat pushing solid ball and 15-s fast pushup were tested by paired samples *t*-test, and the final *P*-value was greater than 0.05, indicating that there was no significant difference, and the controlled experiment could be conducted in this grouping form.

The test results in Table 6 and the test of variance in Table 7 show that the speed and strength levels of the athletes in both groups have improved to a certain extent after the experiment, but the athletes in the experimental group have a particularly significant difference with the control group in the performance of the seated flat pushing solid ball after the experiment (*P* < 0.01); and in the performance of the 15-s fast pushup, although the performance of the athletes in both groups has been improved, there is no significant difference between the performance of the two groups (*P* > 0.05). There was no significant difference between the two groups (*P* > 0.05). This is because the performance of sitting flat pushing solid ball depends entirely on the speed and strength level of the upper limbs of the athletes, while the 15-s fast pushup also has high requirements for muscular endurance, so it cannot fully reflect the speed and strength level of the athletes. In conclusion, the experiment can indeed enhance the speed strength level of the athletes in the experimental group, while the control group does not perform specialized speed strength training, so the speed strength level is not significantly improved.

### 3.3. Comparative Analysis of Punching Techniques of Athletes before and after the Experiment

#### 3.3.1. Comparative Analysis of Punching Speed

This article uses a Sony HDR-CX630E 4K digital camera to calculate the speed of the athlete in the process of punching, and each record is the average speed of three consecutive punches.

The test results in Table 8 and the test of variance in Table 9 show that the average punching speed of the two groups was 6.075 m/s and 6.120 m/s before the start of the experiment, and there was no significant difference between them (*P* > 0.05); after the experiment, the average performance of the experimental group increased to 6.760 m/s, while the performance of the control group increased to 6.190 m/s. It was found that although both groups showed significant changes in performance, the experimental group showed a greater increase in performance.

By comparing the results of the experimental group and the control group after the experiment, it was found that the punching speed of the experimental group had been significantly higher than that of the control group (*P* < 0.01), which indicates that speed strength can indeed effectively improve the punching speed of athletes. Thus, we believe that through the specialized training of speed power in training, it is beneficial to improve the punching speed of the athletes and is an important method to improve the athletes' competition performance.

#### 3.3.2. Comparative Analysis of Punching Power

In this study, the pressure-sensitive sensors were used to test the punching power of the athletes, and the average of three consecutive tests was taken for each test. Due to the limitation of the working principle of the test equipment, only vertical force can be measured, so in the punching power test, the athletes use straight punching method.

The test results in Table 10 and the test of variance in Table 11 show that the average punching power of the two groups was 127 kg and 126 kg before the start of the experiment, and there was no significant difference between them (*P* > 0.05); after the experiment, the average performance of the experimental group increased to 133.5 kg, while the performance of the control group increased to 127.7 kg. It was found that although both groups showed significant changes in performance (*P* < 0.05), the experimental group showed a greater increase in performance.

By comparing the performance of the experimental group with that of the control group, we found that the speed of the experimental group was significantly higher than that of the control group (*P* < 0.01), indicating that speed strength can indeed effectively improve the punching power of athletes. Thus, we believe that through the specialized training of speed power in training, it is beneficial to improve the punching power of the athletes and is an important method to improve the athletes' performance in competition.

### 3.4. Analysis of the Effect of Speed and Power on the Special Hitting Effect of Women's Boxing

#### 3.4.1. The Effect of Speed Power on the Effect of Straight Boxing

In boxing, straight punches are the most direct means of attack and are widely used by high-level boxers in active attack tactics. Straight punches can play the role of testing the opponent and fighting for the initiative of the game. Powerful and fast straight punches will constantly force the opponent to defend and create scoring opportunities. Through the experiments, we found that the speed and power of the punches were significantly improved after the athletes improved their speed and power through special training. This allows the athlete to throw a fast and heavy straight punch when attacking with a straight punch. The speed of the punch reduces the opponent's reaction time and makes it too late to defend or dodge effectively; by increasing the athlete's punching power, the athlete is able to reduce the opponent's possibility of successful defense and create scoring opportunities. In boxing, straight punches are the most direct and effective, fast and heavy straight punches are important for controlling the pace of the game and playing tactics, so that speed and power can largely improve the effectiveness of straight punches, mainly in improving the speed of straight punches to reduce the opponent's reaction time, as well as through more powerful punches to break through the opponent's defense in two ways.

#### 3.4.2. The Effect of Speed and Power on the Effect of Swinging Punches

Unlike the straight punch, the pendulum punch is often used in direct attacks and even more often than the straight punch in defensive counterattacks, mainly because it can effectively reduce the possibility of successful defense of the opponent and create an unexpected tactical effect, creating opportunities for continuous attacks. Through the experiment, we found that the improvement of speed and power can directly improve the punching speed and punching power of athletes, and in the process of defensive counterattack, the punching speed is an important quality indispensable for athletes to make effective counterattack. In the active offense, the swinging punch is combined with the straight punch, and the striking direction is combined with the side, so the swinging punching effect of the athlete is significantly improved in the process of improving the speed power of the athlete. Firstly, because the speed of the athlete's punches is improved, so the athlete is able to counterattack in the shortest possible time after successful defense, when the opponent has no time to react. The offensive intention is not as obvious as the straight punch, so it can greatly improve the chances of scoring. On the other hand, as the athlete's punching power increases, the power of the swinging punch will also increase accordingly, which can form a suppression of the opponent and enable the athlete to quickly complete the change of attacking and defending positions and gain the initiative of the game, which can improve the chances of winning the game.

#### 3.4.3. The Effect of Speed and Power on the Effect of Hook Punching

This is mainly because the success rate of hooks is relatively low, but through the effective use of the hook attack technique, it can also achieve a winning effect, so the hitting effect of hooks is also an important factor in determining the overall competitive level of the athletes. By improving the speed and power of the athlete, the athlete will be able to throw more powerful hooks, which can form an effective suppression of the opponent, and with the speed and power, the speed of the hook is also faster, because the use of the hook itself is less in the game, so through the cooperation of fast punches, opponents often have too little time to react. In boxing matches with big level athletes, the physical confrontation increases and the number of hugs and close range attacks increases, so fast and heavy hooks can effectively hit the opponent hard. So the improvement of speed power can increase the success rate of the hook attack and improve the effectiveness of the use of the hook, and is an important winning factor.

#### 3.4.4. Influence of Speed and Power on the Effect of Combination Punching

Combination boxing has an impact on the control of the rhythm of the game as well as the winner of the game due to the large number of punches and the large change of the striking position. Through the experiment, it was found that the quality of combination boxing strikes was also improved correspondingly after the speed power was increased, which showed that the speed of combination boxing was faster and the strikes were heavier, so the speed power was increased effectively to improve the striking effect of combination boxing.

## 4. Conclusions

1. The athletes improved the test scores of the flat pushing solid ball item through the speed strength special exercises in the experiment and did not improve the scores of the basic movement ability test item, indicating that the experiment did improve the speed strength level of the athletes, but did not have a significant effect on improving the basic movement ability.
2. By comparing the results of the punching speed test items, it was found that with the improvement of speed strength, the punching speed of the athletes in the experimental group was significantly improved, while the athletes in the control group were significantly behind the athletes in the postexperimental test, indicating that the improvement of speed strength could improve the punching speed of the athletes, and the training for speed strength also achieved good results.
3. By comparing the results of the punching power test between the athletes in the experimental group and the control group after the experiment, it was found that the improvement of speed strength significantly improved the punching power level of the athletes in the experimental group, while the athletes in the control group did not gain significant improvement in speed strength, so the improvement level of punching power was much lower than that of the athletes in the experimental group, resulting in a particularly significant difference in the results of the two groups after the experiment. It means that the improvement of speed strength has a positive effect on the punching power of the athletes.
4. With the improvement of the athletes' speed level, the athletes' punching power and punching speed were directly improved, so that the athletes could better play the technical characteristics when attacking with straight punch, swinging punch, and hook technique, and improve the athletes' striking effect, thus increasing the possibility of winning the match.

## Figures and Tables

**Table 1:** Training program for athletes in the experimental group.

Projects	Action	Training volume	Load (small level/medium level/large level)	Break between groups
Preparation activities	Jogging	400 m	—	—
	Barbell squat	8 times × 4 sets	15 kg/20 kg/25 kg	1 min
	Barbell hard pull	8 times × 4 sets	10 kg/15 kg/20 kg	1 min
Traditional strength training	Barbell bench press	8 times × 4 sets	15 kg/20 kg/25 kg	1 min
	Dumbbell upper incline push	12 times × 4 sets	One hand 7.5 kg/10 kg/12.5 kg	1 min
	Dumbbell overhead press	12 times × 4 sets	One hand 5 kg/7.5 kg/10 kg	1 min
Speed strength strengthening training	Dumbbell weighted punching exercises	15 times × 4 sets	2.5 kg	1 min
	Narrow distance jumping pushups	12 times × 4 sets	Self-weight	1 min
	One-handed alternating pushups	12 times × 4 sets	Self-weight	1 min
Finishing activities	Static stretching	10 min	—	—

**Table 2:** Training program for control group athletes.

Projects	Action	Training volume	Load (small level/medium level/large level)	Break between groups
Preparation activities	Jogging	400 m	—	—
	Barbell squat	8 times × 6 sets	15 kg/20 kg/25 kg	1 min
	Barbell hard pull	8 times × 6 sets	10 kg/15 kg/20 kg	1 min
Traditional strength training	Barbell bench press	8 times × 6 sets	15 kg/20 kg/25 kg	1 min
	Dumbbell upper incline push	12 times × 6 sets	One hand 7.5 kg/10 kg/12.5 kg	1 min
	Dumbbell overhead press	12 times × 6 sets	One hand 5 kg/7.5 kg/10 kg	1 min
Finishing activities	Static stretching	10 min	—	—

**Table 3:** Frequency statistics of basic movement ability scores before and after the experiment for the experimental group and the control group.

	Squat		Front and back split-leg squat		Straight knee leg raise		Shoulder joint flexibility		Pushups		Rotational stability	
	Pre-experiment	After the experiment	Pre-experiment	After the experiment	Pre-experiment	After the experiment	Pre-experiment	After the experiment	Pre-experiment	After the experiment	Pre-experiment	After the experiment
(3 points/2 points/1 point/0 point)												
Experimental group	(28/12/0/0)	(30/10/0/0)	(24/16/0/0)	(24/16/0/0)	(21/19/0/0)	(23/17/0/0)	(22/18/0/0)	(22/18/0/0)	(26/14/0/0)	(30/10/0/0)	(19/21/0/0)	(19/21/0/0)
Control group	(29/11/0/0)	(30/10/0/0)	(23/17/0/0)	(24/16/0/0)	(23/17/0/0)	(25/15/0/0)	(23/17/0/0)	(23/17/0/0)	(29/11/0/0)	(32/8/0/0)	(18/22/0/0)	(20/20/0/0)

**Table 4:** Statistics of each test index before the experiment for the experimental group and the control group.

Serial number	Experimental group		Control group	
	Sitting flat pushing solid ball (m)	15 s fast pushups (times)	Sitting flat pushing solid ball (m)	15-s fast pushups (times)
1	5.21	22	5.12	21
2	5.15	24	5.28	25
3	5.36	25	5.03	24
4	5.24	21	5.04	21
5	5.06	20	5.35	23
6	5.37	21	5.10	20
7	5.10	22	5.08	19
8	5.39	23	5.07	18
9	4.98	23	4.96	24
10	4.90	21	5.07	24

**Table 5:** Difference detection of pre-experimental test indexes in the experimental and control groups.

Grouping	Sitting flat pushing solid ball (m)	15-s fast pushups (times)
Experimental group	5.173 ± 0.139	22.000 ± 2.000
Control group	5.140 ± 0.164	21.700 ± 3.114
*P*	0.508	0.719

**Table 6:** Statistics of the test indexes in the experimental group and the control group after the experiment.

Serial number	Experimental group		Control group	
	Sitting flat pushing solid ball (m)	15-s fast pushups (times)	Sitting flat pushing solid ball (m)	15-s fast pushups (times)
1	5.52	24	5.25	23
2	5.39	26	5.3	27
3	5.61	27	5.15	26
4	5.55	23	5.11	13
5	5.61	24	5.44	25
6	6.01	25	5.23	21
7	5.42	27	5.19	21
8	5.59	24	5.17	22
9	5.38	24	5.10	27
10	5.41	24	5.17	25

**Table 7:** Difference detection of postexperimental test indexes in the experimental and control groups.

Grouping	Sitting flat pushing solid ball (m)	15-s fast pushups (times)
Experimental group	5.521 ± 0.164	24.350 ± 1.843
Control group	5.242 ± 0.152	23.300 ± 3.962
*P*	0.002	0.245

**Table 8:** Statistics of punching speed indexes before and after experiments for the experimental group and the control group.

Serial number	Experimental group		Control group	
	Pre-experiment (m/s)	After the experiment (m/s)	Pre-experiment (m/s)	After the experiment (m/s)
1	5.2	6.0	5.3	5.4
2	5.8	6.5	5.6	5.6
3	5.3	6.2	5.5	5.7
4	6.1	7.0	5.9	5.8
5	6.5	6.9	6.7	6.7
6	5.7	6.8	6.1	6.0
7	5.1	5.9	5.5	5.6
8	6.2	7.2	6.1	6.3
9	6.5	7.0	6.0	6.3
10	6.8	7.1	6.3	6.3

**Table 9:** Difference detection of punching speed indexes before and after the experiment for the experimental group and the control group.

Grouping	Experimental group	Control group	*P*
Pre-experimental results (m/s)	6.075 ± 0.578	6.120 ± 0.527	0.508
Postexperimental results (m/s)	6.760 ± 0.458	6.190 ± 0.514	0.001
*P*	0.003	0.027	—

**Table 10:** Statistics of punching power indexes before and after experiments for the experimental group and the control group.

Serial number	Experimental group		Control group	
	Pre-experiment (kg)	After the experiment (kg)	Pre-experiment (kg)	After the experiment (kg)
1	121	130	122	124
2	125	132	123	123
3	126	129	120	122
4	130	133	135	135
5	138	142	136	137
6	134	135	137	138
7	121	129	122	120
8	127	133	125	136
9	124	134	121	127
10	133	137	130	133

**Table 11:** Difference detection of punching power indexes before and after experiments for the experimental group and the control group.

Grouping	Experimental group	Control group	*P*
Pre-experimental results (m/s)	127.000 ± 6.407	126.000 ± 6.308	0.428
Postexperimental results (m/s)	133.500 ± 5.206	127.700 ± 6.626	0.004
*P*	0.001	0.013	—

## Data Availability

All data used in this study can be accessed upon request.
